# Morphophysiological changes in the splenic extracellular matrix of *Leishmania infantum*-naturally infected dogs is associated with alterations in lymphoid niches and the CD4+ T cell frequency in spleens

**DOI:** 10.1371/journal.pntd.0006445

**Published:** 2018-04-20

**Authors:** Aurea Virginia Andrade da Silva, Fabiano Borges Figueiredo, Rodrigo Caldas Menezes, Arthur Augusto Mendes-Junior, Luisa Helena Monteiro de Miranda, Elisa Cupolillo, Renato Porrozzi, Fernanda Nazaré Morgado

**Affiliations:** 1 Laboratório de Pesquisas em Leishmaniose, Instituto Oswaldo Cruz, Fundação Oswaldo Cruz, Rio de Janeiro, Rio de Janeiro, Brazil; 2 Graduate student of the Masters Program in Cellular and Molecular Biology, Instituto Oswaldo Cruz, Fundação Oswaldo Cruz, Rio de Janeiro, Rio de Janeiro, Brazil; 3 Laboratório de Pesquisa Clínica em Dermatozoonoses em Animais Domésticos, Instituto Nacional de Infectologia Evandro Chagas, Fundação Oswaldo Cruz, Rio de Janeiro, Rio de Janeiro, Brazil; Institut national de la recherche scientifique, CANADA

## Abstract

The spleen is one of the main affected organs in canine visceral leishmaniasis (CVL). Disorganization of the splenic white pulp (SWP) has been associated with immunosuppression and disease progression. This study aims to assess structural and cellular changes in the splenic extracellular matrix of dogs with CVL, correlating these changes with the parasite load and clinical signs. Splenic fragments were collected from 41 naturally infected animals for parasite load quantification by quantitative PCR, histopathological analysis and immunohistochemistry for CD3^+^, CD4^+^, and CD8^+^ T cells; CD21^+^ B cells; Ki-67^+^, IFN-γ^+^, and IL-10^+^ cells; and the MMP-9 and ADAM-10 enzymes. Laminin, collagen and fibronectin deposition were also evaluated. The animals were grouped according to the level of SWP organization. SWP disorganization was accompanied by a reduction in the quantity of lymphoid follicles/mm^2^ (p > 0.0001). Animals with moderate to intense SWP disorganization showed more clinical signs (p = 0.021), higher laminin (p = 0.045) and collagen deposition (p = 0.036), higher MMP-9 expression (p = 0.035) and lower numbers of CD4^+^ T cells (p = 0.027) in the spleen than the animals with organized SWP. These data suggest that splenic structure and function are drastically altered and compromised during CVL.

## Author summary

Infected dogs play important roles in the transmission of visceral leishmaniasis. These dogs are considered reservoirs of parasites in urban areas and fail to mount an efficient anti-*Leishmania* immune response. However, the specific immunosuppression profile is not completely understood. In our report, we evaluate and discuss the morphophysiological alterations in the spleens of dogs with visceral leishmaniasis. We found an association between extracellular matrix alterations and a failure to control the parasite load. We suggest a role for these alterations in hindering an immune response that is otherwise able to control the parasite load, thereby leading to disease progression. Our research contributes to the current knowledge of the immunopathology of canine visceral leishmaniasis.

## Introduction

In Brazil, visceral leishmaniasis is caused by *Leishmania infantum*, and the domestic dog is the main urban reservoir[1]. Additionally, dogs have been used as models for the study of human disease[2] because disease progression in dogs is similar to that in humans[3].

Concerning the immune response in canine visceral leishmaniasis (CVL), susceptible animals have a remarkably attenuated humoral and cellular immune response against the parasite, resulting in the appearance of clinical signs[2]. Although the cytokine expression profile has also been associated with disease resistance or progression to CVL[4], the data regarding cytokine expression in the spleen remain controversial[1,5,6].

The spleen is the key organ responsible for removing damaged and senescent cells from blood circulation. The adaptive immune responses against the pathogens captured from the blood begin in this organ[7]. The composition of the spleen is based on two structures: the red pulp and the white pulp, an area rich in T and B lymphocytes. Additionally, cells that are highly specialized in antigenic presentation are found in this organ. The white pulp exhibits an organization in which it is wrapped around central arterioles, which are branches of the artery[7]. Multiple molecules, namely, laminin, fibronectin and collagen, are important proteins that constitute the basal and interstitial membranes of this organ and are fundamental to the structuring and maintenance of the white pulp, contributing to the upkeep of cellular compartmentalization. These proteins also contribute to the cellular communication and transport of cytokines and chemokines through structures known as sinusoids and conduits, which comprise type IV collagen, laminin and reticular fibroblasts[8–10]. Differences in the localizations of extracellular matrix (ECM) molecules in the spleen suggest that the ECM plays a role in the compartmentalization of immune cells to their respective niches, and clearly, future analyses of ECM animal models require the consideration of possible immunological defects[10].

The spleen is among the main organs affected by CVL and is responsible for the immune response to systemic infection; however, knowledge on the pathogenic mechanisms involved is limited. Splenic microarchitecture disruption in infected dogs has been associated with fibrosis and disease progression[11,12]. The increased deposition of laminin, fibronectin and collagen in the livers of naturally infected dogs, with a concomitant decrease in T lymphocytes and an increase in the parasite load, has been described elsewhere[13]. Still, the structural changes of the splenic ECM are accompanied by reductions in the mRNA expression levels of chemokines and their receptors[14]. These authors have suggested that the failure to express these molecules may lead to deficient leukocyte migration, hampering the development of an efficient immune response. Although metallopeptidases (MMP-2 and MMP-9), which are enzymes that degrade ECM compounds, have already been demonstrated in the sera of naturally infected dogs[15], their activities in tissues, particularly in the spleens of infected dogs, have not been evaluated. We hypothesized that changes in the organization of splenic white pulp (SWP) could be accompanied by alterations in ECM molecule deposition, metallopeptidase activity and lymphocyte distribution, thereby affecting the immune response and resulting in failure to control the parasite, especially during the final stages of the disease. Thus, the aim of the present study was to examine alterations to splenic ECM compounds through the analysis of collagen, laminin and fibronectin deposition and metallopeptidase expression (MMP-9, ADAM-10) in groups of animals showing different degrees of SWP organization. Additionally, we aimed to describe and compare the distributions and quantities of T and B lymphocytes in their segregated areas, proliferation markers (Ki-67) and cytokine expression (IFN-γ and IL-10) in these groups. Herein, the disorganized SWP from dogs naturally infected with *L*. *infantum* showed a higher deposition of ECM compounds, namely, laminin and collagen, and higher MMP-9 *in situ* expression than the organized SWP. These alterations were associated with reductions in lymphocyte niches and the frequency of CD4^+^ cells.

## Methods

### Ethics statement

The animals included in this study were *L*. *infantum*-naturally infected dogs that were destined for euthanasia as recommended by the politics of the Brazilian Ministry of Health and after all owners of the dogs had provided formal written consent. The samples were collected during necropsies conducted by veterinarians from the Laboratório de Pesquisa Clínica em Dermatozoonoses em Animais Domésticos (LAPCLIN-DERMZOO–INI/FIOCRUZ) approved by Comitê de Ética em Uso de Animais (CEUA—Fiocruz) under the license LW-54/13 and according to the Brazilian Law 11794/08 and Sociedade Brasileira de Ciência em Animais de Laboratório (SBCAL).

### Animals and clinical evaluation

Forty-one dogs from Barra Mansa- (Rio de Janeiro, Brazil), obtained from a convenience sampling, diagnosed with CVL were included in this study. Later, the animals were grouped according to the level of SWP organization. The primary diagnosis was performed by Centro de Controle de Zoonoses da Secretaria Municipal de Barra Mansa using the CVL DPP test (Bio-Manguinhos-FIOCRUZ) as the screening test and ELISA (EIE–Leishmaniose Visceral Canina Bio-Manguinhos) as the confirmatory test. In addition, the infection was confirmed by parasite isolation, and all animals were associated with positive cultures in NNN/Schneider's biphasic medium at 25°C.

The animals included in the study were negative for the most common hemoparasitoses with Fuller Kit (Eurovet—Babesia canis) and Snap 4DX Plus Test (IDEXX -Anaplasma/Ehrlichia/Lyme/Heartworm). All dogs with coinfections (hemoparasitosis and leishmaniasis) were excluded from this study.

Clinical evaluations were performed by two veterinarians according to the clinical score adapted elsewhere[16,17]. Shortly, six common clinical signs (dermatitis, onychogryphosis, keratoconjunctivitis, the body condition, alopecia and lymphadenopathy) were scored on a semiquantitative scale from 0 (absent) to 3 (severe). Body condition was classified as 0 (Ideal: easily palpable ribs with minimal fat around, waist easily seen from above and evident abdominal silhouette), 1 (Thin: ribs easily palpable and may be visible without palpable fat, the top of the lumbar region is visible, prominent pelvic bones, silhouette of waist and abdomen apparent), 2 (Very thin: Ribs, lumbar and pelvic bones are easily visible, absence of palpable fat, evidence of other bony prominences and minimal muscle loss) and 3 (Extremely thin: All bony structures are prominent and in evidence at a distance, no discernible body fat and severe loss of muscle mass). None of the evaluated animals showed obesity. The sum of the values was used to determine the final clinical classification as low (0–2), moderate (3–6) or high (7–18) score. After clinical examination, euthanasia was conducted by veterinarians from the LAPCLIN-DERMZOO by intravenously administering 1.0 ml/kg 1.0% Thiopental (Thiopentax, Cristália). After the absence of a corneal reflex due to deep anesthesia was detected, 10 ml of 19.1% potassium chloride was intravenously administered (Isofarma). During necropsy, tissue samples from the spleen were collected into sterile DNA-free polypropylene tubes and frozen at -20°C until further use.

### DNA extraction

Total DNA was extracted from approximately 10 mg of each spleen sample. The DNA extraction was performed using the QIAmp DNA Mini kit (Qiagen, CA, USA), which included an initial phase of digestion with 20 μl of proteinase K (20 mg/mL) for 1 hour at 56°C. The DNA was dissolved in 50 μl of tris EDTA buffer (AE buffer) and quantified with the NanoDrop spectrophotometer (Thermo Scientific, USA).

### Determination of *Leishmania* load by quantitative polymerase chain reaction (qPCR)

The parasite loads in the spleen samples were estimated by quantitative PCR (qPCR) as previously described by Cavalcanti and collaborators[17]. HPRT primers (Supplementary S1 Table) were used to normalize the concentrations of canine DNA in each sample. To quantify the parasite load, primers (S1 Table) described by Prina and collaborators[18] were used to amplify a product corresponding to the small subunit ribosomal RNA (ssrRNA, multicopy gene). The qPCR reactions were run with the Step One equipment (Applied Biosystems, Molecular Probes, Inc.) using the detection system Power SYBR Green Master Mix (Applied Biosystems, Molecular Probes, Inc.). Total purified DNA (100 ng) in 2 μl was added to a final PCR reaction volume of 20 μl containing 1X Power SYBR Green and 300 nM of each primer for HPRT or 500 nM of each primer for ssrRNA PCR. qPCR was performed with an activation step at 95°C for 10 minutes, followed by 40 cycles of denaturation and annealing/extension (95°C for 15 seconds, 60°C for 1 minute and 68°C for 30 seconds). A melt curve stage was performed for each specific amplification analysis (95°C for 15 seconds, 60°C for 1 minute and 95°C for 15 seconds). All reactions were performed in duplicate for each target, and both targets were run in the same plate for the same sample. Quantifications of peripheral blood mononuclear cells (PBMC) from non-infected dogs and *L*. *infantum* promastigotes (MCAN/BR/2007/CG-1) were performed using a cell counter (Z1 COULTER COUNTER, Beckman Coulter, Fullerton, CA, USA), and total DNA was extracted from 1.0 x 10^6^ PBMCs and 1.0 x 10^7^ promastigotes. Standard curves for HPRT and ssrRNA genes were prepared using serial 10-fold dilutions from 10^−2^ to 10^7^ of total purified DNA. The animals were grouped as high or low parasite burden (cutoff: 5.5 x 10^4^ parasites/10^6^ host cells) as described by Cavalcanti et al[17].

### Histopathology

The spleen fragments were fixed in 10% formalin, embedded in paraffin and cut into 5-μm-thick sections that were mounted on microscope slides. The sections were stained with hematoxylin and eosin and examined by light microscopy (Nikon Eclipse E400 –Tokyo, Japan). Structural changes to spleen lymphoid tissues were analyzed as previously described[19]. The parameters analyzed were as follows: the presence of granulomas and the degree of the structural organization of the white pulp (1, *organized*–the presence of a distinct periarteriolar lymphocyte sheath, germinal center, mantle zone and marginal zone; 2, *slightly disorganized*–the presence of either hyperplastic or hypoplastic changes leading to a loss in the definition of any region of the white pulp; 3, *moderately disorganized*–evident white pulp with poorly individualized or indistinct regions; and 4, *intensely disorganized*–a follicular structure that was barely distinct from the red pulp and T cell areas). The number of lymphoid follicles was determined as lymphoid follicles/mm^2^ of tissue in tissues sections using Nikon ACT-1 software version 2.62 (Nikon). Well-formed granulomas were characterized by the presence of epithelioid cells and well-established limits. Collagen deposits were quantified in picrosirius red-stained tissue using ImageJ 1.48v software (NIH, USA). Since the parameters evaluated did not differ infected dogs presenting organized SWP from those of uninfected dogs, animals presenting organized SWP were considered as the reference for comparisons between groups.

### Immunohistochemistry

Immunohistochemistry was based on the method reported by Morgado and collaborators[20]. Briefly, spleen fragments frozen in OCT resin (Sakura) were cut into 3–5 μm-thick sections and mounted onto microscope slides (silanized slides; DakoCytomation, Carpinteria, CA, USA). The slides were fixed in acetone PA (Merck, Darmstadt, Germany) and subjected to hydration, endogenous peroxidase blockage (peroxidase blocking reagent; Dako) and nonspecific staining blockage (0.4% BSA; Sigma, USA). The specimens were then incubated with primary antibodies directed against CD3^+^, CD4^+^, CD8^+^, CD21^+^, IFN-γ^+^, IL-10^+^ (Serotec), Ki-67^+^ (eBioscience), laminin, fibronectin, ADAM-10 (Abcam) or MMP-9 (Serotec), followed by incubation with the Labelled Polymer (Envision System-HRP, Dako). Aminoethyl carbazole (AEC kit; Invitrogen) was used as the substrate-chromogen system, and the slides were counterstained with Mayer’s hematoxylin (Sigma). The slides were examined under a light microscope (Zeiss), and the number of marked cells/mm^2^ tissue in the red pulp was determined. Two blinded readers evaluated the slides. Laminin and fibronectin deposits were quantified using ImageJ 1.48v software (NIH, USA), and the results are presented as the percentage of the marked area. Primary antibody suppression was used as the negative control reaction.

### Statistical analysis

The SPSS program for Windows, version 16 (SPSS Inc., Chicago, IL, USA) was used for statistical analysis. The Kolmogorov-Smirnov test was used to evaluate the Gaussian distributions of the variables. The data were analyzed using Student’s t-test for variables with parametric distributions and the Mann-Whitney test for variables with nonparametric distributions. Correlations were determined using Spearman’s rank correlation coefficient. The data are reported as the mean and standard error of the mean (SEM) or and the median and minimum and maximum values. Non-numerical data were analyzed in 2 x 2 contingency tables with Fisher’s exact test using Prism software (GraphPad Prism version 6.01). P-value < 0.05 was considered significant.

## Results

### Lymphoid follicles/ tissue is lower in animals with disorganized splenic white pulp (SWP) than in animals with well-structured splenic stroma

Considering the 41 animals diagnosed with CVL included in this study, the main clinical signs observed were onychogryphosis (79.4%), followed by dermatitis (67.6%), loss of body condition (41.2%), alopecia (38.2%), lymphadenomegaly (23.5%) and keratoconjunctivitis (23.5%) (S1 Fig and S2 Table). The animals were classified into 3 groups based on the clinical score: 1-low score (N = 13, 31.7%); 2-moderate score (N = 15; 36.6%); and 3-high score (N = 13; 31.7%).

Based on histopathological analysis of the spleen, the white pulp was classified as organized SWP (OR, n = 3, 7.31% and Fig 1A), slightly disorganized SWP (SD, n = 8, 19.51% and Fig 1B), moderately disorganized SWP (MD n = 15, 36.6% and Fig 1C) and intensely disorganized SWP (ID; n = 15, 36.6% and Fig 1D). We observed that the higher the level of SWP disorganization was, the smaller the number of lymphoid follicles would be (P-value = 0.0001) (Fig 1E). The animals with MD-ID SWP showed higher clinical scores (median 6.0; range 0 to 12.0) than the animals with OR-SD SWP (clinical score: median 1.0; range 0 to 8.0 P-value = 0.021) (Fig 1F).

**Fig 1:** Degrees of disorganization of the splenic white pulp in dogs naturally infected with *Leishmania infantum*. (A) Organized splenic white pulp: the white pulp has a distinct periarteriolar lymphocyte sheath, germinal center, mantle zone and marginal zone; (B) slightly disorganized splenic white pulp: the white pulp shows a decrease in the definition of any white pulp region; (C) moderately disorganized splenic white pulp: the white pulp is evident, but its regions are poorly defined or indistinct; (D) intensely disorganized white pulp; the follicular structure is barely distinct from the red pulp or T cell areas. Scale bar = 100 μm. Hematoxylin and eosin. (E) Lymphoid follicle number in the splenic white pulp. (F) The clinical scores of the evaluated dogs. Mann-Whitney test. OR-SD = animals with organized to slightly disorganized splenic white pulp. MD-ID = animals with moderately to intensely disorganized splenic white pulp.

The analysis of the granuloma number/mm^2^ of splenic tissue revealed that only 6 dogs showed well-formed granulomas (n = 6; median 3.83 × 10^6^; minimum-maximum 4,6100–20,300,000 parasites/10^6^ cells), and this finding was accompanied by a higher parasite burden compared to the samples that did not show well-formed granulomas (n = 35; median 5.26 × 10^5^; minimum-maximum 145–6,970,000 parasites/10^6^ cells, P-value = 0.039).

### The deposition of the extracellular matrix components is associated with the disorganization of the splenic white pulp

Most of the dogs analyzed in this study (n = 30, 73.2%) showed moderate to intense SWP disorganization. We hypothesized that this disorganization was associated with a modification to ECM molecule expression. In this context, the expression of laminin, fibronectin and collagen were analyzed by immunohistochemistry (Fig 2A–2M).

**Fig 2:** The extracellular matrix components in the spleens of naturally infected dogs with *L*. *infantum*. (A) Negative control (suppression of primary antibody). (B-D) Fibronectin deposition. Note that the deposition is well distributed throughout the splenic tissue and within the follicle (D). (E) Negative control (suppression of primary antibody). (F-G) The deposition of laminin is homogenous throughout the red pulp; however, laminin expression is delimited around the marginal zone of the white pulp (H). (I) Negative control. (J-L) Collagen deposition in the red pulp and (M) in one granuloma. A, B, D, F, H, I, J and M show the animals with organized splenic white pulp. C, E, G and L show the animals with disorganized splenic white pulp. Magnification: (A-H) 100x; Scale bar: 100 μm and (I-M) 400x; Scale bar: 25 μm. A-H: Immunohistochemistry—aminoethyl carbazole. I-M: Picrosirius red. (N) fibronectin deposition/area; (O) laminin deposition/area; (P) collagen deposition/area. Mann-Whitney test. OR-SD = animals with organized to slightly disorganized splenic white pulp. MD-ID = animals with moderately to intensely disorganized splenic white pulp.

Fibronectin deposition was more abundant in the red pulp and in the intrafollicular than laminin deposition (Fig 2C and 2D, respectively). In general, the deposition of laminin was less intense in the intrafollicular region than in the red pulp (Fig 2H). In the MD-ID group, the laminin deposition assumed an irregular distribution. For example, in the follicle delimitation, laminin deposition was discontinuous and less intense in the animals with moderately to severely disorganized SWP than in the animals with organized to slightly disorganized SWP. We did not observe differences in fibronectin deposition when the groups were compared (Fig 2M). Higher laminin and collagen deposition in dogs with moderately to intensely disorganized SWP were observed (Fig 2O and 2P and S3 Table, P-value = 0.045 and 0.036, respectively). To determine whether the alterations in laminin deposition were accompanied by alterations in fibronectin deposition, we correlated these data and observed a positive correlation between laminin and fibronectin deposition (P-value = 0.043; r^2^ = 0.393 and S2A Fig).

### Metallopeptidase-9 expression is higher in dogs with disorganized splenic white pulp than in dogs with organized spleen

We investigated whether MMP-9 and ADAM-10, two peptidases associated with matrix remodeling, could be altered in animals presenting different degrees of SWP disorganization by immunohistochemistry (Fig 3C and 3D). MMP-9 expression was higher in animals with MD-ID SWP than in animals with OR-SD SWP (P-value = 0.035) (Fig 3E and S3 Table). No significant differences were observed for ADAM-10 expression (P-value>0.05) (Fig 3F and S2 Table).

**Fig 3:** Deposition of MMP-9 and ADAM-10 during the extracellular matrix remodeling process. The dogs with disorganized splenic white pulp showed higher MMP-9, but not ADAM-10, expression than the dogs with organized splenic white pulp. (A-B) Negative controls (suppression of primary antibody) (C) Immunostaining of MMP-9. (D) Immunostaining of ADAM-10. Both immunostaining procedures were performed in the red pulp. (E) MMP-9 expression. (F) ADAM-10 expression. Immunohistochemistry of the red pulp—aminoethyl carbazole. Magnification: 400x, Scar bar: 25 μm. OR-SD = animals with organized to slightly disorganized splenic white pulp. MD-ID = animals with moderately to intensely disorganized splenic white pulp.

### The CD4^+^ cell number is lower in the disorganized spleen than in the organized spleen

To examine the lymphocyte subpopulations of the disorganized spleen, CD4^+^, CD8^+^ and CD21^+^ cells were quantified in the red pulp (Fig 4A–4J) since no individual lymphoid structure can be observed in intensely disorganized tissue. The CD4^+^ T cell number was lower in the MD-ID animals than in the OR-SD animals (P-value = 0.027, Fig 4K and S3 Table). No differences in the numbers of CD8^+^ and CD21^+^ cells were evident between the groups (Fig 4L and 4M and S3 Table) (P-value>0.05). To verify whether associations between the cellular profile and extracellular molecule or metallopeptidase alterations were present, we correlated these data and observed positive correlations between collagen deposition and CD21^+^ cells (P-value = 0.008 and r^2^ = 0.418; S2B Fig) and between CD21^+^ cells and MMP-9 expression (P-value = 0.010 and r^2^ = 0.401; S2C Fig). We also evaluated IFN-ɣ^+^- and IL-10^+^-expressing cells. Although no differences were evident between groups, a correlation between IFN-ɣ^+^ and IL-10^+^ expression was observed (P-value = 0.0074 and r^2^ = 0.412) (Fig 4N and 4O and S2D Fig).

**Fig 4:** CD4^+^, CD8^+^ and Ki-67 ^+^ expression and cytokines/mm^2^ splenic tissue of dogs naturally infected with *L*. *infantum*. (A-B) Negative control (suppression of primary antibody). Immunostaining of (C-D) CD3^+^, (E) CD4^+^, (F) CD8^+^, (G) CD21^+^, (H) Ki-67^+^ proliferating, (I) IFN-ɣ^+^ and (J) IL-10^+^ cells. Magnification in A and C: 100x; Magnification in B and D-J: 400x. Scale bar = 25 μm. (L) CD4^+^ T cells/mm^2^. (M) CD8^+^ T cells/mm^2^. (N) CD21^+^ B cells/mm^2^. (O) Expression of IFN-ɣ/mm^2^; (P) IL-10/mm^2^; (Q) KI-67^+^ cells/mm^2^. Mann-Whitney test. OR-SD = animals with organized to slightly disorganized splenic white pulp. MD-ID = animals with moderately to intensely disorganized splenic white pulp.

### Association of the morphophysiological alterations and parasite load

Because the dogs were naturally infected and because the parasite load and splenic histopathological alterations were noted as markers of infection/disease progression, as described elsewhere[5,12], we examined the associations between the parasite load and splenic histopathological alterations. According to Cavalcanti[17], we grouped the dogs as follows: 1-Low parasite load and organized SWP (LOW/OR), 2- Low parasite load and disorganized SWP (LOW/DS) and 3-High parasite load and disorganized SWP (HIGH/DS) (Fig 5). When these groups were compared, a low lymphoid follicle number (Fig 5A) and high laminin deposition (Fig 5B) were detected even in dogs with low parasite loads. Collagen deposition (P-value = 0.041) and MMP-9 expression (P-value = 0.035) were higher in the LOW/DS and HIGH/DS groups than in the LOW/OR group (Fig 5D and 5E). No differences in ADAM-10 expression were evident between the groups (Fig 5F). Furthermore, no differences in fibronectin deposition or in the numbers of CD8^+^, CD21^+^ and Ki-67^+^ cells/mm^2^ were evident (P-value>0.05) (Fig 5C and 5H–5J). However, a lower CD4^+^ cells/mm^2^ red pulp value was observed in LOW/DS dogs than in LOW/OR dogs (Fig 5G). In addition, the number of CD4^+^ cells/mm^2^ red pulp of the HIGH/DS animals was similar to that of the LOW/DS animals (P-value>0.05). However, the reduction in size and the atrophy in both the lymphoid periarteriolar sheath and lymphoid follicles in the spleens from dogs with high parasite loads and similar numbers of CD4^+^ cells in the red pulp favor the hypothesis that SWP disorganization contributes to difficulties in cell migration (Fig 5G, the raw data are shown in the S4 Table).

**Fig 5:** Association between the histopathological analysis and parasite burden. (A) Lymphoid follicles, (B) laminin deposition, (C) fibronectin deposition, (D) collagen deposition, (E) MMP-9 expression, (F) ADAM-10 expression, (G) CD4^+^ cells, (H) CD8^+^ cells, (I) CD21^+^ cells and (J) Ki-67^+^ cells. P-value < 0.05 was considered significant. Mann-Whitney test. Low/OR = low parasite burden and organized to slightly disorganized splenic white pulp. Low/DS = low parasite burden and moderately to intensely disorganized splenic white pulp. High/DS = high parasite burden and moderately to intensely disorganized splenic white pulp.

## Discussion

Herein, alterations in histology, ECM compounds, metallopeptidase expression and CD4^+^ cell quantity were detected in the spleens of dogs naturally infected with *Leishmania infantum*. SWP microarchitecture disorganization was observed in most of the animals (N = 30, 73.2%). The disorganized SWP showed a reduction in the size and number of lymphoid follicles and the periarteriolar sheath, as well as a low number of CD4 ^+^ lymphocytes in the red pulp, suggesting that T and B lymphocytes were not migrating to their specific sites and/or were beginning apoptosis. A reduction in spleen cellularity has already been demonstrated in a murine model of experimental infection with *L*. *infantum*[21]. The spleen is a secondary lymphoid organ that contains segregated areas of T and B lymphocytes, which favors the antigenic presentation and activation of these cells. An absence of or reduction in lymphocytes in their respective areas can lead to an activation deficit that contributes to the failure to control the parasite load. We observed low numbers of CD4 ^+^ cells in the animals with moderate to intense SWP disorganization. In CVL, the spleen shows a marked reduction in the gene expression levels of several cytokines, chemokines and their receptors[16,17]. In particular, a reduction in CXCL13 is associated with atrophy and lymphoid follicle disorganization[6]. We observed that the majority of animals with low parasite loads already had SWP disorganization and low numbers of CD4^+^ T cells, with concomitantly high laminin expression.

Dogs with disorganized SWP, even those with low parasite loads, showed high laminin, collagen and MMP-9 expression. This high expression of ECM molecules can be caused by the intense inflammation occurring at the beginning of infection[5,15]. The increase of MMP-2 and MMP-9 in the sera of dogs with visceral leishmaniasis has been previously demonstrated[15,22]. Thus, in our study, we found that MMP-9 expression was higher in dogs with disorganized SWP than in dogs with organized SWP. Moreover, MMP-9 expression was more intense in dogs with high parasite burdens and disorganized SWP. In this context, as observed in cardiomyopathy, the expression levels of metalloproteinases, such as MMP-9, MMP-3 and MMP-10, produced by activated macrophages[23] can be positively regulated during this initial inflammatory process, leading to alterations in the degradation of collagen, laminin and fibronectin, to facilitate the migration of inflammatory cells to the site of infection, consequently modifying the organization of the SWP. MMP-9 plays a role in the orientation of cell migration, with ECM degradation mainly affecting type IV collagen, vascular remodeling and the inflammatory process[15,24,25].

The increased deposition of ECM components has been described in the livers of dogs[13] and in the murine thymus and lymph node[8] and has been correlated with an increased parasite load, suggesting that the deposition of fibronectin and laminin might be responsible for the success of the infection[13]. Fibronectin degradation can generate peptide fragments, which bind to receptors in macrophages, hampering the activation and function of these cells. Furthermore, the changes in the deposition of these components may reflect the inflammatory and degenerative processes, which is ultimately important in the dissemination of the parasite[19].

On the other hand, we cannot exclude the possibility that the parasite has direct effects on the ECM molecules. In this context, the direct effect of *L*. *amazonensis* promastigotes on an *in vitro* collagen matrix has been previously demonstrated[26]. When an animal is inoculated, the promastigotes are exposed to the dermis, which comprises ECM, growth factors and resident cells[27]. To establish the infection, promastigotes must overcome the obstacles presented by the dermal ECM, which may affect the tissue and thereby contribute to pathogenesis[27,28]. However, herein, we evaluated dogs with chronic infections, and the effects of amastigotes on ECM remain unknown.

In the liver, laminin and fibronectin expression were correlated with the parasite burden and disease progression in dogs naturally infected with *L*. *infantum (syn*. *L*. *chagasi)*, suggesting that these molecules were important to the invasion of *Leishmania* parasites[13]. We found an association between high laminin expression and ECM remodeling. Moreover, our results showed that high laminin expression was evident even when the parasite load was still low, suggesting that laminin could play roles in all stages of infection.

Another metallopeptidase evaluated in this study was ADAM-10, and ADAM-10 expression was detected in all evaluated groups. No differences in ADAM-10 expression were observed between the studied groups, which suggests that although this disintegrin is involved in type IV collagen degradation[23,25], in the lymphoid follicle ontogeny[29,30] and in the regulation and maintenance of the lymphoid architectures of secondary lymphoid organs[29,31], ADAM-10 expression is not associated with SWP disorganization in the animals included in this study.

Animals with disorganized SWP presented high laminin deposition and low amounts of CD4^+^ cells. In thymic tissue, O'campo and collaborators[32] have reported that laminin is associated with the premature migration of CD4^+^ T and CD8^+^ T lymphocytes. In this context, CD4^+^ cells are leaving the spleen via mechanisms not yet known. In dogs with high parasite loads, we observed that the number of CD4^+^ cells in the red pulp was similar to that in dogs with organized white pulp; however, atrophy of the lymphoid periarteriolar sheath and lymphoid follicles was evident. We suggest that CD4^+^ cells in advanced infection may not have been able to migrate to their specific compartments within the white pulp due to the low expression levels of chemokines, cytokines and their receptors[6,14,21,33,34] or due to alterations in the distributions of splenic conduits. Additional experiments should be performed to confirm this hypothesis.

Granuloma formation, which is an efficient immune response for controlling parasite burden in visceral leishmaniasis, is one parameter for evaluations of the cell-mediated immune response[35]. In the present study, we observed the presence of well-formed granulomas only in 6 animals; however, in murine experimental infections, a marked infectious granulomatous reaction, which involved Kupffer cells, in the liver led to parasite load control[36,37]. Herein, the parasite burdens in the dogs with well-formed granulomas were higher than in the dogs in which granulomas were not observed. These data suggest a delay/deficit in the formation of an efficient immune response by the evaluated dogs. In acute phase of experimental *Leishmania infantum*-infection in macaque model, there was a strong Th1 response, and parasite load could be controlled in blood, bone marrow, lymph nodes and liver but not in the spleen where the parasite burden remained constantly [38]. During the chronic phase, the immune response converted to an IL-10-dominated environment in the spleen [38]. Herein, the studied dogs were naturally infected, and probably were in the chronic phase, which could explain the absence of differential IL-10 expression when the groups were compared. Altogether, the data presented herein support the conclusion that the disorganization of the splenic microarchitecture is a frequent alteration in the evaluated dogs, suggesting that the splenic structure and function are drastically altered and compromised during CVL. These alterations to ECM compounds and immune cells might consequently lead to immunosuppression and severe disease.

## Supporting information

S1 Fig The frequency of clinical signs in naturally infected dogs with *Leishmania infantum*. Forty-one naturally infected animals were included in this study. The most common clinical signs were onychogryphosis (79.4%) and dermatitis (67.6%), followed by weight loss (41.2%), alopecia (38.2%), lymphadenopathy (23.5%) and keratoconjunctivitis (23.5%).
(TIF)

S2 Fig Correlations between the extracellular matrix (ECM) components, cell subpopulations and parasite burden. (A) Laminin and fibronectin, (B) CD21^+^ cells and collagen deposition, (C) CD21^+^ cells and MMP-9 expression, (D) IL-10 and IFN-ƴ expression, (E) CD8^+^ cells and parasite burden. Spearman correlation.
(TIF)

S1 Table Target genes and primers designed for DNA quantification and parasite load determination. S, sense; AS, antisense; bp, base pairs.
(DOCX)

S2 Table Clinical data collected from each dog. (DOCX)

S3 Table Frequency of cells, metallopeptidases and extracellular matrix compounds in the spleens of dogs naturally infected with *L. infantum* according to spleen organization. *P-value = 0.045; **P-value = 0.036; P-value = ***0.022; P-value = ****0.027.
(DOCX)

S4 Table Frequency of cells, metalloproteases and extracellular matrix compounds according to splenic organization and parasite burden in dogs naturally infected with *L. infantum*. *P-value = 0.005; **P-value = 0.041; P-value = ***0.035; P-value = ****0.0021.
(DOCX)

S5 Table Raw data from the dogs naturally infected with *L. infantum* that were evaluated in this study. a: 1 = Low; 2 = High. b: 1 = Organized; 2 = Slightly disorganized; 3 = Moderately disorganized; 4 = Intensely disorganized. c: 1 = Low parasite burden/Organized splenic white pulp; 2 = Low parasite burden/disorganized splenic white pulp; 3 = High parasite burden/disorganized splenic white pulp. d: 1 = Yes; 2 = No.
(DOCX)
